The article "1, 25-D3 Protects From Cerebral Ischemia by Maintaining BBB Permeability via PPAR-γ Activation" was retracted in 2023. Reasons: unreliable data; unreliable results or conclusions; concerns about the images.

# 1, 25-D_3_ Protects From Cerebral Ischemia by Maintaining BBB Permeability via PPAR-γ Activation

**DOI:** 10.3389/fncel.2018.00480

**Published:** 2018-12-17

**Authors:** Ting Guo, Yanqiang Wang, Yuanfang Guo, Shuguang Wu, Weiwei Chen, Na Liu, Yu Wang, Deqin Geng

**Affiliations:** ^1^Department of Neurology, Xuzhou Medical University, Xuzhou, China; ^2^Department of Neurology, The Affiliated Hospital of Xuzhou Medical University, Xuzhou, China; ^3^Department of Neurology, The Affiliated Hospital of Weifang Medical University, Weifang, China; ^4^Department of Respiratory Medicine, Ganyu District People’s Hospital, Lianyungang, China; ^5^Department of Anesthesiology, The Second Affiliated Hospital of Zhejiang University School of Medicine, Hangzhou, China; ^6^Department of Neurology, The Central Hospital of Xuzhou, Xuzhou, China

**Keywords:** BBB permeability, 1, 25-D_3_, MCAO/R, PPARγ, NF-κB, inflammation, BDNF

## Abstract

The blood-brain barrier (BBB) is a physical and biochemical barrier that maintains cerebral homeostasis. BBB dysfunction in an ischemic stroke, results in brain injury and subsequent neurological impairment. The aim of this study was to determine the possible protective effects of 1, 25-dihydroxyvitamin D_3_ [1, 25(OH)_2_D_3_, 1, 25-D_3_, vit D] on BBB dysfunction, at the early stages of an acute ischemic brain injury. We analyzed the effects of 1, 25-D_3_ on BBB integrity in terms of histopathological changes, the neurological deficit, infarct size and the expression of brain derived neurotrophic factor (BDNF), in a middle cerebral artery occlusion/reperfusion (MCAO/R) rat model. BBB permeability and the expression of permeability-related proteins in the brain were also evaluated by Evans blue (EB) staining and Western blotting respectively. To determine the possible mechanism underlying the role of 1, 25-D_3_ in BBB maintenance, after MCAO/R, the rats were treated with the specific peroxisome proliferator-activated receptor gamma (PPARγ) inhibitor GW9662. Supplementation with 1, 25-D_3_ markedly improved the neurological scores of the rats, decreased the infarct volume, prevented neuronal deformation and upregulated the expression of the tight junction (TJ) and BDNF proteins in their brains. Furthermore, it activated PPARγ but downregulated neuro-inflammatory cytokines such as nuclear factor kappa-B (NF-κB) and tumor necrosis factor-α (TNF-α), after MCAO/R. Taken together, 1, 25-D_3_ protects against cerebral ischemia by maintaining BBB permeability, upregulating the level of BDNF and inhibiting PPARγ-mediated neuro-inflammation.

## Introduction

Stroke is a common neurological disorder accompanied by a high risk of disability and mortality (Ludewig et al., 2013; Deng et al., 2016). Ischemic stroke can disrupt the blood-brain barrier (BBB), and induce brain edema, inflammation and neuronal injury, all of which cause severe structural and functional deterioration (Chen et al., 2016; Wicha et al., 2017; Zhang H. T. et al., 2017). Although the recombinant tissue-type plasminogen activator (rt-PA) has a certain therapeutic effect on ischemic stroke as a thrombolytic agent, its clinical use is limited due to the narrow therapeutic window and its adverse effects (Zhang Q. Y. et al., 2017). Therefore, it is necessary to identify novel drugs against ischemic stroke and elucidate their underlying mechanisms of action (Li et al., 2014; Lin et al., 2015; He et al., 2016, 2017; Janyou et al., 2017; Liu et al., 2017; Miah et al., 2017).

The article "1, 25-D3 Protects From Cerebral Ischemia by Maintaining BBB Permeability via PPAR-γ Activation" was retracted in 2023. Reasons: unreliable data; unreliable results or conclusions; concerns about the images.

As the name suggests, BBB acts as a cordon between the brain and blood vessels, and consists of endothelial cells, pericytes, astrocytes, neurons and the extracellular matrix (Beard et al., 2011; Pillai et al., 2013; Venkat et al., 2017; Wu et al., 2018). Increasing evidence indicates that BBB impairment is a key pathological manifestation of ischemic stroke, for e.g., brain edema and hemorrhage, development of the inflammatory cascade and secondary ischemic injury (Gu et al., 2013; Zhang Q. Y. et al., 2017). Therefore, repairing and maintaining the BBB is potentially neuro- and vaso-protective in stroke and requires attenuating the decrease in vascular endothelial cell tight junction (TJ) proteins such as occludin, claudin-5 and ZO-1, as well as controlling inflammatory reactions (Xin et al., 2012; Wang et al., 2015; Huang et al., 2017; Shi et al., 2017). The transcription factor peroxisome proliferator-activated receptor gamma (PPARγ), is a promising therapeutic target in animal models of stroke, traumatic brain injury, Alzheimer’s disease (AD) and Parkinson’s disease (PD), by maintaining BBB function and decreasing brain inflammation, oxidative stress and neuronal injury (Liu et al., 2018). A recent study showed that the activation of PPAR-γ downregulated nuclear factor kappa-B (NF-κB) and its downstream inflammatory response pathway in cerebrovascular diseases such as stroke (Huang et al., 2016). PPARγ activation is also known to upregulate the brain-derived neurotrophic factor (BDNF) in neurodegenerative diseases such as AD and PD (Aleshin et al., 2013; Falcone et al., 2015). The BDNF is a member of the neurotrophin family and is frequently downregulated in rodent models of stroke, indicating that low BDNF levels are closely associated with the increased risk of stroke. However, the pathways mediating the effects of PPARγ on BBB integrity and function are largely unknown. Several studies have shown that 1, 25-dihydroxyvitamin D_3_ (1, 25-D_3_) inhibits inflammation, reactive oxygen species (ROS) production and infiltrate circulating immune cells after stroke (Wang et al., 2000; Durk et al., 2012, 2014; Nissou et al., 2014). Deficiency of 1, 25-D_3_ aggravated stroke injury in a rat model, while supplementing with 1, 25-D_3_ restored brain function (Won et al., 2015). Although the post-ischemic neuroprotective effects of 1, 25-D_3_ are well documented, its potential effects on BBB after ischemic cerebral injury and the underlying mechanisms are still unknown.

The article "1, 25-D3 Protects From Cerebral Ischemia by Maintaining BBB Permeability via PPAR-γ Activation" was retracted in 2023. Reasons: unreliable data; unreliable results or conclusions; concerns about the images.

Recent studies have highlighted a potential therapeutic cross talk between 1, 25-D_3_ and PPARγ in myocardial infarction and ischemia reperfusion-induced acute kidney injury (Kapil et al., 2013). We therefore hypothesized that 1, 25-D_3_ maintains BBB integrity by upregulating BDNF levels, possibly via the PPARγ-dependent anti-inflammatory pathway. Our findings show that 1, 25-D_3_ plays an important role in preserving the BBB.

## Materials and Methods

### Animals and Housing

Male Sprague-Dawley (SD) rats (250–280 g) were obtained from the Experimental Animal Center of Xuzhou Medical University, and kept in a temperature-controlled (22 ± 2°C) room with a 12 h light/ dark cycle (lights on at 6:00 a.m.) and 55 ± 10% humidity. All experiments were conducted as per the guidelines of the Institutional Animal Care and Use Committee of China, and approved by the Ethics Committee for the Use of Experimental Animals at Xuzhou Medical University.

### Establishment of the Middle Cerebral Artery Occlusion/Reperfusion (MCAO/R) Rat Model

The SD rats were randomized into the following five groups: Sham-operated, middle cerebral artery occlusion/reperfusion (MCAO/R), vehicle (dimethyl sulfoxide, DMSO), MCAO/R+1, 25-D_3_ and MCAO/R+1, 25-D_3_+GW9662 and treated accordingly. The 1, 25-D_3_ (Macklin, China) was dissolved in 2% DMSO and administered intravenously (5 mg/kg/ml) 30 min before surgery. GW9662 (Bingham, UK) was dissolved in 2% DMSO and administered intravenously (0.3 mg/kg) to the MCAO/R+1, 25-D_3_+ GW9662 group rats, 60 min before surgery. The MCAO/R model was established as described previously (Zong et al., 2017). Briefly, the rats were anesthetized with intraperitoneal ketamine (60 mg/kg) and xylazine (5 mg/kg) after overnight fasting. The right common carotid artery (CCA), right internal carotid artery (ICA) and right external carotid artery (ECA) were exposed through a ventral midline neck incision, and the branches of ECA were ligatured. A 4-0 nylon monofilament with a rounded tip (Guangzhou Jialing Biotechnology Co. Ltd., China) was inserted along the CCA into the ICA until a slight resistance was detected. Ninety minutes after MCAO, the monofilament was pulled out, followed by a reperfusion at 6 h, 12 h, 24 h, 3 days and 5 days post-MCAO. The same surgery was performed in the sham group rats, without filament insertion.

The article "1, 25-D3 Protects From Cerebral Ischemia by Maintaining BBB Permeability via PPAR-γ Activation" was retracted in 2023. Reasons: unreliable data; unreliable results or conclusions; concerns about the images.

### Assessment of Neurological Deficit

Neurological function was evaluated at 6 h, 12 h, 24 h, 3 days and 5 days after reperfusion using a modified Neurological Severity Scale (mNSS; Chen et al., 2001). It includes a battery of motor, sensory, reflex and balance tests similar to the contralateral neglect tests applied to humans. Neurological function was graded on a scale of 0–18 (normal score 0 and maximal deficit score 18). All rats had sufficient time to acclimatize themselves to the testing environment before surgery, and a score of 0 in the mNSS test was indicative of MCAO/R (Zong et al., 2017).

### Infarct Volume Measurement

The rats were anesthetized with ketamine (60 mg/kg, i.p) and xylazine (5 mg/kg, i.p) at the afore-mentioned time points post-MCAO/R, and 2 mm coronal slices were cut. The tissues were stained with a 2% solution of 2,3,5-triphenyltetrazolium chloride (TTC; Sigma, St. Louis, MO, USA) in a phosphate buffered saline (PBS) at 37°C, and then fixed with paraformaldehyde. Areas that stained deep red represented the undamaged area after MCAO/R, while the white colored regions indicated the infarct area. Infarct sizes were quantified using ImageJ software, and the percentage of relative infarction volume (RIVP) was calculated by the formula: RIVP = IVA/TA × 100%, where IVA and TA are the infarcted and total areas of the coronal sections respectively.

### Hematoxylin-Eosin (HE) Staining

The rats were anesthetized as described, and then sequentially perfused with 0.9% NaCl and 4% paraformaldehyde. The brains were dissected and embedded in paraffin, and 5 mm slices were cut with a microtome. The brain slices were stained by hematoxylin-eosin (HE; Sigma, St. Louis, MO, USA) as per standard protocols.

### Measurement of BBB Permeability

Evans blue (EB) was used as a tracer to measure the permeability of the BBB as described previously. Briefly, 2% EB (2 ml/kg, Sigma, St. Louis, MO, USA) was injected intravenously into the rats and allowed to circulate for 24 h. The rats were then anesthetized and transcardially perfused with 0.9% NaCl. The brains were removed, split into the left and right hemispheres, and the right hemispheres were immersed in formamide (10 ml/kg, Sigma, St. Louis, MO, USA) at 60°C for 24 h. The tissues were then centrifuged (5,000 rpm, 10 min) at 4°C, and the absorbance of the supernatants was measured at 632 nm. The EB content was calculated from its standard curve as a measure of the BBB permeability change. EB extravasation in the peri-ischemic cortex was also observed using a DMI 6000 digital microscope (Leica, Germany).

The article "1, 25-D3 Protects From Cerebral Ischemia by Maintaining BBB Permeability via PPAR-γ Activation" was retracted in 2023. Reasons: unreliable data; unreliable results or conclusions; concerns about the images.

### Immunofluorescent Staining

On first day after reperfusion, the animals were anesthetized and transcardially perfused with 0.9% NaCl and then 4% paraformaldehyde. The fixed brains were extracted and further perfused with 4% paraformaldehyde overnight and then dehydrated in 30% sucrose until shrinkage occurred. The cerebral peri-ischemic cortices were cut into consecutive slices (20 μm each) and washed with PBS. The slices were first incubated with the blocking solution (0.1% Triton X-100 in 0.1 M PBS, 10% bovine serum albumin, pH 7.6) for 2 h and then overnight with anti-occludin (1:100, Abcam, USA) and anti-claudin-5 (1:100, Thermo Fisher Scientific, Rockford, IL, USA) antibodies at 4°C. After washing with PBS, the tissues were incubated with the secondary antibodies and counterstained with 4′,6-diamidino-2-phenylindole (DAPI, Beyotime, China). The stained sections were observed under a DMI 6000 digital microscope (Leica, Germany).

### Western Blotting

The rats were euthanized with a ketamine (60 mg/kg, i.p) and xylazine (5 mg/kg, i.p) injection, and their brains were dissected. The peri-ischemic cortical proteins were extracted by homogenizing the thawed tissues in a RIPA lysis buffer containing the protease and phosphatase inhibitors and centrifuged at 14,000 rpm for 20 min at 4°C. Protein concentration was measured using a BCA assay kit (Thermo Fisher Scientific, Rockford, IL, USA). Equal amounts (60 μg) of protein per sample were separated by SDS-PAGE before transferring to PVDF membranes (Millipore, USA). Non-specific binding was blocked with 5% skim milk for 90 min, and the membranes were then incubated overnight with rabbit anti-PPARγ (1:1,000, Abcam, USA), anti-NF-κB (1:1,000, Abcam, USA), anti-β-actin (1:5,000, ABclonal, China), anti-occludin (1:1,000, Abcam, USA), anti-claudin-5 (1:500, Thermo Fisher Scientific, Rockford, IL, USA), anti-tumor necrosis factor-α (anti-TNF-α; 1:2,000, Abcam, USA) and anti-BDNF (1:1,000, Abcam, USA) antibodies at 4°C. After washing with TBST (0.1%) and incubating with secondary antibodies, the immuno-reactive bands were visualized by chemiluminescence using an ECL kit (Beyotime, China). The specific bands were analyzed using ImageJ software.

### Statistical Analysis

All data were expressed as Mean ± SEM. The Student’s *t*-test was used to compare the two groups, and a one-way analysis of variance (ANOVA) was used for multiple comparisons. All statistical analyses were conducted using a GraphPad Prism 5. *P*-values < 0.05 were considered statistically significant.

The article "1, 25-D3 Protects From Cerebral Ischemia by Maintaining BBB Permeability via PPAR-γ Activation" was retracted in 2023. Reasons: unreliable data; unreliable results or conclusions; concerns about the images.

## Results

### 1, 25-D_3_ Improves Neurological Performance in Rats After Stroke

To determine the effects of 1, 25-D_3_ on a brain injury, a mNSS was used to evaluate the neurological score of the rats at 6 h, 12 h, 24 h, 3 days and 5 days after reperfusion. The MCAO/R rats showed poor neurological function compared to the sham-operated and compared with DMSO-treated groups, treatment with 1, 25-D_3_ significantly improved neurological performance at all time points after reperfusion, with an optimum effect at 24 h post-surgery, while GW9662 reversed the protective effect of 1, 25-D_3_ at 24 h, 3 days and 5 days after reperfusion (Figure 1, ***P < 0.001, ^##^*P* < 0.01, ^#^*P* < 0.05 and ^ &^*P* < 0.05). Taken together, 1, 25-D_3_ improved the neurological deficit in MCAO/R rats.

**Figure 1:** Pre-treatment with 1, 25-D_3_ (Vit D) improved MCAO/R-induced neurological impairment. The modified Neurological Severity Scale (mNSS) scores in the different groups were evaluated at 6 h, 12 h, 24 h, 3 days and 5 days after reperfusion. Data are represented as Mean ± SEM, *n* = 6, ***P < 0.001 vs. sham group, ^##^*P* < 0.01 vs. DMSO group, ^#^*P* < 0.05 vs. DMSO group, ^&^*P* < 0.05 vs. 1, 25-D_3_ group. MCAO/R, middle cerebral artery occlusion/reperfusion; DMSO, dimethyl sulfoxide; PPAR-γ, peroxisome proliferator-activated receptor-gamma; 1, 25-D_3_, 1, 25-dihydroxyvitamin D_3_; GW9662, inhibitor of PPAR-γ.

### Pretreatment With 1, 25-D_3_ Ameliorated Early Brain Injury After MCAO/R

The infarct volumes at the different time points post-reperfusion were measured by TTC staining (Figure 2, ***p < 0.001, ^###^*P* < 0.001, ^&&^*P* < 0.01 and ^&^*P* < 0.05), which indicated the absence of any cerebral ischemic infarct in the sham-operated group but significant ischemic injury in the MCAO/R model group. No significant differences were observed between the infarct sizes of the vehicle (DMSO) and MCAO/R groups. However, pre-treatment with 1, 25-D_3_ significantly reduced the infarct volume, which was reversed by GW9662 treatment at 24 h, 3 days and 5 days after reperfusion. Therefore, 1, 25-D_3_ pre-treatment protected against cerebral MCAO/R injury. In addition, since the smallest infarct volume in the treated animals was observed 24 h after reperfusion, we selected this time point for subsequent experiments.

**Figure 2:** 1, 25-D_3_ (Vit D) decreased the infarct volume. **(A–E)** Rat brains were sliced and stained with 2,3,5-triphenyltetrazolium chloride (TTC) at the 6 h, 12 h, 24 h, 3 days and 5 days after MCAO/R and the percentage of relative infarct volume was calculated. Data are represented as Mean ± SEM, *n* = 6, ***P < 0.001 vs. sham group, ^###^*P* < 0.001 vs. DMSO, ^&&^*P* < 0.01 vs. 1, 25-D_3_ group, ^&^*P* < 0.05 vs. 1, 25-D_3_ group. MCAO/R, middle cerebral artery occlusion/reperfusion; DMSO, dimethyl sulfoxide; PPAR-γ, peroxisome proliferator-activated receptor-gamma; 1, 25-D_3_, 1, 25-dihydroxyvitamin D_3_; GW9662, inhibitor of PPAR-γ.

The article "1, 25-D3 Protects From Cerebral Ischemia by Maintaining BBB Permeability via PPAR-γ Activation" was retracted in 2023. Reasons: unreliable data; unreliable results or conclusions; concerns about the images.

### 1, 25-D_3_ Reduced the Deformation of Nerve Cells

The histopathological effects of 1, 25-D_3_ after MCAO/R was examined by HE staining. As shown in Figure 3, no obvious pathological changes occurred in the cortices of the sham-operated rats and the neurons were well-arranged with abundant cytoplasm (Figure 3A). In contrast, the brains of the MCAO/R and vehicle treated rats showed both serious histological damage in the ischemic zone, as well as degenerative changes reflected by irregularly arranged neurons, deep coloration, and increased gaps around the neurons (Figures 3B,C, ***P < 0.001). Pre-treatment with 1, 25-D_3_ markedly improved the histological integrity of the cortex compared to that of the untreated rats. In addition, deep coloration was observed in a small number of cells with clearer borders (Figure 3D, ^###^*P* < 0.001). Treatment with GW9662 however, reversed the neuro-protective effects of 1, 25-D_3_ (Figure 3E, ^&&^*P* < 0.01). Thus, 1, 25-D_3_ has a potent long-term neuroprotective function against IR injury, which is abrogated by GW9662.

**Figure 3:** 1, 25-D_3_ (Vit D) protected against neuronal injury induced by cerebral ischemic reperfusion 24 h after MCAO/R. **(A–E)** Representative pictures of hematoxylin-eosin (HE) stained cerebral cortex. **(F)** Number of positively stained cells in the cerebral cortex was analyzed using the ImageJ software (400× magnification). Data are represented as Mean ± SEM, *n* = 6, ***P < 0.001 vs. sham group, ^###^*P* < 0.001 vs. DMSO group, ^&&^*P* < 0.01 vs. 1, 25-D_3_ group. MCAO/R, middle cerebral artery occlusion/reperfusion; DMSO, Dimethyl sulfoxide; 1, 25-D_3_, 1, 25-dihydroxyvitamin D_3_; GW9662, inhibitor of PPAR-γ.

### 1, 25-D_3_ Protected Against MCAO/R-Induced BBB Permeability

To evaluate whether 1, 25-D_3_ also protected the BBB, brain sections were stained with EB (Figures 4A,B), and its extravasated amount was measured. As shown in Figure 4C, MCAO induced significant extravasation of EB compared to the sham-operated group, in the 24 h following reperfusion. Pre-treatment with 1, 25-D_3_ significantly reduced EB extravasation (Figure 4C, ***P < 0.001, ^###^*P* < 0.001, ^&&^*P* < 0.01), while GW9662 reversed the effects of 1, 25-D_3_ on BBB permeability. These results indicated that 1, 25-D_3_ protected MCAO/R rats from the ischemic damage on BBB permeability and this effect was abrogated by GW9662.

The article "1, 25-D3 Protects From Cerebral Ischemia by Maintaining BBB Permeability via PPAR-γ Activation" was retracted in 2023. Reasons: unreliable data; unreliable results or conclusions; concerns about the images.

**Figure 4:** 1, 25-D_3_ (Vit D) restores blood-brain barrier (BBB) integrity impaired by ischemic reperfusion. **(A)** Evans blue (EB)-stained brains 24 h following MCAO/R. **(B)** EB stained (red) brain sections (original magnification 400×). **(C)** Levels of extravasated EB (μg/g of brain tissue). Data are represented as Mean ± SEM, *n* = 6, ***P < 0.001 vs. the sham group, ^###^*P* < 0.001 vs. DMSO group, ^&&^*P* < 0.01 vs. 1, 25-D_3_ group. MCAO/R, middle cerebral artery occlusion/reperfusion; DMSO, dimethyl sulfoxide; 1, 25-D_3_, 1, 25 dihydroxyvitamin D_3_; PPAR-γ, peroxisome proliferator-activated receptor-gamma; GW9662, inhibitor of PPAR-γ.

### 1, 25-D_3_ Pre-treatment Restored the Expression Levels of Tight Junction Proteins in MCAO/R Rats

To further confirm the effect of 1, 25-D_3_ on BBB permeability, we also analyzed the expression levels of the TJ proteins occludin and claudin-5, which play important roles in BBB integrity and permeability. MCAO/R significantly weakened *in situ* occludin and claudin-5 expression 24 h after reperfusion, compared to the control group. The levels of both proteins, recovered after treatment with 1, 25-D_3_ and were markedly downregulated by GW9662 (Figures 5A,B). These results were confirmed by Western blotting (Figures 5C–E, ***P < 0.001, ^###^*P* < 0.001, ^#^*P* < 0.05, ^&&^*P* < 0.01 and ^&^*P* < 0.05). Thus, 1, 25-D_3_ protected the BBB after stroke by inhibiting degradation of the TJ.

**Figure 5:** 1, 25-D_3_ (Vit D) protected against tight junction (TJ) degradation induced by cerebral ischemic reperfusion 24 h after MCAO. **(A,B)** *In situ* expression of claudin-5 (green), occludin (red) and 4′,6-diamidino-2-phenylindole (DAPI; blue) in the peri-infarct region of sham-operated, MCAO/R, DMSO, 1, 25-D_3_ and GW9662 groups (400× magnification 400). **(C–E)** Western blots showing the expression levels of occludin and claudin-5 in the ischemic cortical tissue. Data are represented as Mean ± SEM, *n* = 6, ***P < 0.001 vs. sham group, ^###^*P* < 0.001 vs. DMSO group, ^#^*P* < 0.05 vs. DMSO group, ^&&^*P* < 0.01 vs. 1, 25-D_3_ group. ^&^*P* < 0.05 vs. 1, 25-D_3_ group. MCAO/R, middle cerebral artery occlusion/reperfusion; 1, 25-D_3_, 1, 25-dihydroxyvitamin D_3_; DMSO, dimethyl sulfoxide; PPAR-γ, peroxisome proliferator-activated receptor-gamma; GW9662, inhibitor of PPAR-γ.

### 1, 25-D_3_ Pre-treatment Suppressed the MCAO/R-Induced Inflammatory Response by Activating PPARγ

Since inflammation is the major pathogenic basis of BBB injury, we evaluated the effects of 1, 25-D_3_ on the levels of inflammatory mediators. In addition to activating PPARγ, 1, 25-D_3_ significantly reduced the levels of the inflammatory cytokine TNF-α and the pro-inflammatory transcription factor NF-κB in the MCAO/R rats. Moreover, 1, 25-D_3_ increased the expression of BDNF. However, GW9662 reversed these effects of 1, 25-D_3_ (Figures 6A–E, ***P < 0.001, ^###^*P* < 0.001 **P < 0.01, ^##^*P* < 0.01, ^&&^*P* < 0.01 and ^&^*P* < 0.05. Thus, 1, 25-D_3_ exerted an anti-inflammatory effect on the MCAO/R rats by modulating the PPARγ/TNF-α/NF-κB axis and increasing BDNF expression levels.

The article "1, 25-D3 Protects From Cerebral Ischemia by Maintaining BBB Permeability via PPAR-γ Activation" was retracted in 2023. Reasons: unreliable data; unreliable results or conclusions; concerns about the images.

**Figure 6:** 1, 25-D_3_ (Vit D) pre-treatment suppressed the MCAO/R-induced inflammatory response by activating PPAR-γ. **(A)** The representative image of western-blot analysis for PPAR-γ, TNF-α, NF-κB and BDNF. **(B–E)** PPAR-γ, TNF-α, NF-κB and BDNF expression levels in the brain tissues of different groups were analyzed by Western blotting. Data are represented as mean ± SEM, *n* = 6, ***P < 0.001 vs. sham group, **P < 0.01 vs. sham group, ^###^*P* < 0.001 vs. DMSO, ^##^*P* < 0.01 vs. DMSO, ^&&^*P* < 0.01 vs. 1, 25-D_3_ group, ^&^*P* < 0.05 vs. 1, 25-D_3_ group. MCAO/R, middle cerebral artery occlusion/reperfusion; 1, 25-D_3_, 1, 25-dihydroxyvitamin D_3_; DMSO, dimethyl sulfoxide; GW9662, inhibitor of PPAR-γ; NF-κB, nuclear factor kappa-B; TNF-α, tumor necrosis factor-α; BDNF, brain derived neurotrophic factor.

## Discussion

We investigated the effects of 1, 25-D_3_ on reperfusion-induced BBB disruption in a MCAO/R rat model and found that pre-treatment with this 1, 25-D_3_ protected the rats from neurological deficits, reduced the infarct volume and prevented neuronal injury after MCAO/R. Mechanistically, 1, 25-D_3_ activated PPARγ, inhibited the pro-inflammatory TNF-α and NF-κB, and restored the levels of TJ proteins, thereby protecting against a BBB breakdown. In conclusion, we have shown for the first time that pre-treatment with 1, 25-D_3_ protected BBB integrity after cerebral IR injury by activating the PPARγ-mediated anti-inflammatory effects.

It was observed that the neurons necrotize and die rapidly after ischemic stroke in the infract core, while those in the surrounding region (i.e., the penumbra area) die several hours to days after IR onset. This points to a narrow time window wherein the injured neurons can be rescued from autophagy and necrosis, and therefore be a plausible target for treating stroke (Pengyue et al., 2017). We found that the infarcted region in the brains of MCAO/R animals made up approximately 30% of the whole brain area (Figure 2). Pre-treatment with 1, 25-D_3_ significantly reduced the infarct area and neuronal injury (Figures 2, 3), with an optimum therapeutic effect seen 24 h after MCAO/R (Figures 1, 2).

The article "1, 25-D3 Protects From Cerebral Ischemia by Maintaining BBB Permeability via PPAR-γ Activation" was retracted in 2023. Reasons: unreliable data; unreliable results or conclusions; concerns about the images.

The BBB separates the brain tissues from the blood (Zhu et al., 2015; Janyou et al., 2017; Zhang et al., 2018). Inflammatory molecules, mechanical or hypoxic damage of vascular endothelium and the destruction of the basal lamina by matrix metalloproteinases and excito-toxic amino acids, can degrade the BBB after stroke, leading to vasogenic edema, an influx of toxic substances and neuro-inflammation (Li et al., 2014; Liu et al., 2014; Ji et al., 2015; Miah et al., 2017; Shiraishi et al., 2017). Changes in the BBB function and its basement membrane integrity after ischemic injury lead to the loss of neural tissue and increased para-cellular permeability, which induces intracranial hypertension and brain death. Therefore, in order to stop the progression of IR injury, it is vital to maintain the BBB. In the present study, pre-treatment with 1, 25-D_3_ reduced the damage to the BBB integrity caused by MCAO/R injury (Figures 4A,B) and markedly decreased EB leakage (Figure 4C). To our knowledge, this is the first study to report a protective role of 1, 25-D_3_ against MCAO/R-induced injury.

The structural integrity and function of the BBB is the result of highly selective TJs between the endothelial cells in the central nervous system (CNS) vessels, which is primarily made of the membrane-associated accessory proteins occludin and claudin-5 (Liu et al., 2015, 2017; Zhu et al., 2015; He et al., 2017; Zhang et al., 2018). To further address the underlying mechanisms of the protective effects of 1, 25-D_3_ against MCAO/R, we determined the levels of TJ proteins after the IR injury. Pre-treatment with 1, 25-D_3_ upregulated claudin-5 and rescued occludin loss, which was instrumental in maintaining BBB integrity in the ischemic rat brains (Figure 5). Although 1, 25-D_3_ is a secosteroid hormone and regulates the expression of neurotrophic factors, its most important function in the cerebral tissues is that of an anti-inflammatory agent (Nissou et al., 2014; Guo et al., 2016; Alam et al., 2017). Deficiency in 1, 25-D_3_ is a determinant causative factor of several neurodegenerative and neuropsychiatric disorders (Nissou et al., 2014).

The NF-κB pathway is known to trigger the inflammatory response. During the early period of ischemia reperfusion injury, TNF-α is released by neurons, glia cells and endothelial cells that are activated in response to ischemia reperfusion. This is followed by the synthesis of IL-8 and cell adhesion molecules and the secretion of selectins and β2 integrin, which regulate the levels of adhesion molecules and initiate leukocyte recruitment and invasion, thus leading to further BBB disruption (Huang et al., 2016; Chen et al., 2018). The NF-κB pathway also regulates the expression of TJ proteins in various neurological diseases (Fu et al., 2014; Zhai et al., 2017; Zhang et al., 2018). We found that 1, 25-D_3_ decreased NF-κB activation in the MCAO/Rep rat model, which supported our hypothesis that 1, 25-D_3_ protects BBB integrity against cerebral IR injury via its anti-inflammatory effects. Further studies are needed to validate the involvement of this pathway in BBB disruption post IR injury.

The article "1, 25-D3 Protects From Cerebral Ischemia by Maintaining BBB Permeability via PPAR-γ Activation" was retracted in 2023. Reasons: unreliable data; unreliable results or conclusions; concerns about the images.

NF-kB activation is regulated by the PPAR transcription factors (Deng et al., 2016). PPARγ, the most studied PPAR isoform, has shown the most potent neuroprotective effects in different models of neurodegenerative disorders such as I/R-induced brain injury and AD (Zhao et al., 2006; Zolezzi et al., 2014; Wu et al., 2016; Chen et al., 2018). Consistent with this, co-treatment of the MCAO rats with 1, 25-D_3_ and a PPARγ inhibitor blocked the protective effects of the former, on brain injury (Grommes et al., 2013; Wang et al., 2016; Chen et al., 2018). In this study, GW9662 also reversed the effects of 1, 25-D_3_ on cerebral IR injury, thereby indicating that 1, 25-D_3_ ameliorated inflammation in the MCAO/R rats via the NF-κB and PPARγ signaling pathways. In addition, 1, 25-D_3_ upregulated BDNF, which is known to exert a neuroprotective effect against brain injuries such as cerebral ischemic neuronal damage, in the MCAO/R rats (Figure 6). Several studies have shown that BDNF decreases the infarct volume and improves neurological outcomes following cerebral injury. Consistent with those findings, 1, 25-D_3_ significantly decreased NF-κB and TNF-α and increased the expression levels of BDNF in the MCAO/R rats.

In summary, our findings demonstrated that 1, 25-D_3_ protected rats against MCAO/R injury by preventing BBB disruption through the activation of the anti-inflammatory PPARγ pathway and upregulation of BDNF.

## Author Contributions

TG and YanW wrote the main manuscript text. TG, YanW, YG, SW, WC, NL and YuW performed the experiments and data analyses. DG designed the study and revised the manuscript. All authors approved the final version of the manuscript.

## Conflict of Interest Statement

The authors declare that the research was conducted in the absence of any commercial or financial relationships that could be construed as a potential conflict of interest.
